RETRACTED

# High glucose promotes annulus fibrosus cell apoptosis through activating the JNK and p38 MAPK pathways

**DOI:** 10.1042/BSR20190853

**Published:** 2019-07-08

**Authors:** Lizhen Shan, Di Yang, Danjie Zhu, Fabo Feng, Xiaolin Li

**Affiliations:** 1 Department of Endocrinology and Metabolism, The Second Affiliated Hospital, Zhejiang University School of Medicine, Hangzhou 310009, Zhejiang, China; 2 Department of Orthopaedic Surgery, Zhejiang Provincial People’s Hospital, Hangzhou 310014, Zhejiang, China; 3 People’s Hospital of Hangzhou Medical College, Hangzhou 310014, Zhejiang, China

**Keywords:** annulus fibrosus, apoptosis, high glucose, intervertebral disc degeneration, JNK, p38 MAPK

## Abstract

Diabetes mellitus (DM) is an important risk factor of intervertebral disc degeneration. A high glucose niche-mediated disc cell apoptosis is an implicate causative factor for the spine degenerative diseases related with DM. However, the effects of a high glucose niche on disc annulus fibrosus (AF) cell apoptosis and the potential signaling transduction pathway is unclear. The present study is to investigate the effects of high glucose on disc AF cell apoptosis and the role of two potential signaling pathways in this process. Rat AF cells were cultured in baseline medium or medium with different concentrations (0.1 and 0.2 M) of glucose for 3 days. Flow cytometry was used to assess the degree of apoptosis. Activity of caspase 3/9 was evaluated by chemical kit. Expression of pro-apoptotic and anti-apoptotic molecules was analyzed by real-time polymerase chain reaction and Western blot. In addition, activity of the C-Jun NH_2_-terminal kinases (JNK) pathway and p38 mitogen-activated protein kinase (MAPK) pathway was evaluated by Western blot. Compared with the control group, high glucose culture increased cell apoptosis ratio and caspase-3/9 activity, up-regulated expression of bax, caspase-3, cleaved caspase-3 and cleaved PARP, and down-regulated expression of bcl-2 in a glucose concentration-dependent manner. Additionally, high glucose culture increased expression of the p-JNK and p-p38 MAPK in a concentration-dependent manner. Further results showed that inhibition of the JNK or p38 MAPK pathway attenuated the effects of high glucose on AF cell apoptosis. Together, high glucose promoted disc AF cell apoptosis through regulating the JNK pathway and p38 MAPK pathway in a glucose concentration-dependent manner.

## Introduction

Diabetes mellitus (DM) is a common public health problem around the world. There are two types of DM (type 1 DM and type 2 DM) with approximately 90% of DM patients are type 2 DM [1]. Accumulating evidence has shown that DM is a crucial effecter in the progression of intervertebral disc degeneration [2–6]. The morbidity of disc degeneration is much higher in DM patients than that in non-DM patients [7]. Hence, further investigating the mechanism through which DM induces disc degeneration is necessary to develop effective treatments for DM-associated disc degeneration.

RETRACTED

Intervertebral disc is a cartilaginous structure connecting two adjacent vertebral bones. It is consisted of three closely connected parts: cartilage endplate (CEP), nucleus pulposus (NP) and annulus fibrosus (AF) [8]. AF is a type of lamellar, fibrocartilaginous structure that confines the central NP tissue [9]. Cells of the AF tissue originate from mesenchyme and present many features similar to fibroblasts and chondrocytes [10,11]. AF cells help to maintain the structural integrity through synthesizing and secreting normal and adequate extracellular matrix, whereas some intrinsic and extrinsic pathways activated by the detrimental pathological factors often induce AF cell apoptosis [12,13]. In the previous animal disc degeneration models [12,14], the number of apoptotic AF cells is significantly increased, indicating that AF cell apoptosis is promoted and involved in the progression of disc degeneration.

The high glucose niche in DM patients often increases oxidative stress reaction-associated substrates, which is a potential biochemical pathway behind the DM-associated disease [15,16]. Previously, some studies have reported that a high glucose environment significantly promotes senescence of disc NP cells, notochordal cells and AF cells [17–19]. Moreover, several studies have showed that a high glucose environment induces apoptosis of disc CEP cells and notochordal cells [20,21]. However, few studies have observed the effects of a high glucose environment on disc AF cell apoptosis.

In the present study, we mainly aimed to observe the effects of different concentrations of high glucose on disc AF cell apoptosis, and investigate the role of the p38 mitogen-activated protein kinase (MAPK) pathway and C-Jun NH_2_-terminal kinases (JNK) pathway. Flow cytometry was used to assess the degree of apoptosis. Activity of caspase 3/9 was evaluated by chemical kit. Expression of pro-apoptotic and anti-apoptotic molecules was analyzed by real-time polymerase chain reaction (PCR) and Western blot. In addition, activity of the JNK pathway and p38 MAPK pathway was evaluated by Western blot.

## Materials and methods

### AF cell isolation and culture

The experiment procedure was fully approved by the Animal Ethical Committee of Zhejiang University and performed in the Animal Experimental Center of the Second Affiliated Hospital of Zhejiang University. After lumbar discs were separated from thirty-eight female Sprague–Dawley rats (270–280 g, 8–9 weeks old) that were purchased from the Animal Center of Zhejiang Provincial People’s Hospital. AF tissue samples were obtained after removing the attached soft tissues. Then, AF cells were isolated following the subsequent two-step digestion (0.25% collagenase type I for 30–40 min and 0.25% trypsin for 5–10 min). The isolated AF cells were put in the DMEM/F12 medium supplemented with 10% fetal bovine serum (FBS, Gibco, USA) under standard culture conditions (95% air, 5% CO_2_, 37°C). After going through two passages, AF cells were used in each designed experiment. Briefly, AF cells were cultured in the baseline culture medium (control cells) or medium with two concentrations of glucose (0.1 and 0.2 M) for 3 days.

RETRACTED

### Flow cytometry assay

AF cell apoptosis was evaluated using the Annexin V-fluorescence isothiocyanate (FITC)/propidium iodide (PI) Apoptosis Detection Kit (Beyotime, China). Briefly, after AF cells were cultured in the conditioned medium, both the attached AF cells and the floated AF cells were collected. Then, they were re-suspended in 195 μl Annexin V-FITC binding buffer, followed by incubation with 5 μl Annexin V-FITC and 10 μl PI for 20 min in the dark environment. Finally, the prepared AF cells were analyzed by a flow cytometry machine.

### Caspase-3 and caspase-9 activity measurement

The activity of caspase-3 and caspase-9 was detected using Caspase-3/9 Activity Detection Kit (Beyotime, China). Briefly, after AF cells were cultured in the conditioned medium, both the attached AF cells and the floated AF cells were collected. Then, the supernatant samples in each group were used to analyze the caspase-3/9 activity according to the manufacturer’s instructions.

### Real-time PCR assay

After AF cells were cultured in conditioned medium, they were washed with sterile phosphate buffer solution (PBS) for two times. Total RNA was extracted with TRIzol reagent (Invitrogen, USA) and reverse-transcribed into cDNA samples using a Quantscript RT Kit. Real-time PCR was performed on the reaction system containing cDNA, primers (Table 1) and SYBR Green PCR Master Mix (Applied Biosystems, USA). GAPDH was used as an internal control. The reaction conditions were as follows: 1 cycle of 3 min at 95°C, followed by 35 cycles of 10 s at 95°C, 15 s at 56°C, 30 s at 72°C, and 1 cycle of 3 min at 72°C. The relative expression of investigated genes was calculated using the method of 2^−ΔΔ*C*^_T_.

**Table 1:** Primers of target genes

Gene	Forward (5′-3′)	Reverse (5′-3′)
*GAPDH*	CCGCGAGTACAACCTTCTTG	TGACCCATACCCACCATCAC
*Bcl-2*	GGGGCTACGAGTGGGATACT	GACGGTAGCGACGAGAGAAG
*Bax*	CCAGGACGCATCCACCAAGAAG	GCTGCCACACGGAAGAAGACC
*Caspase 3*	GTACAGAGCTGGACTGCGGTATTG	AGTCGGCCTCCACTGGTATCTTC

RETRACTED

### Western blot assay

After AF cells were cultured in the conditioned medium, they were washed with sterile PBS for two times. Total protein samples were extracted by RIPA solution (Beyotime, China), and then quantified using a BCA Protein Assay Kit (Beyotime, China). After protein samples were separated by sodium dodecyl sulfate/polyacrylamide gel electrophoresis (SDS/PAGE), they were transferred on to the polyvinylidene fluoride (PVDF) membranes (Beyotime, China). Then, the PVDF membranes were sequentially immunostained with primary antibodies (GAPDH: Abcam, ab181602; cleaved caspae-3: Cell Signaling Technology, #9664; Cleaved PARP: Cell Signaling Technology, #94885; JNK: Cell Signaling Technology, #9255; p-JNK: Cell Signaling Technology, #9252; p38 MAPK: Abcam, ab31828; p-p38 MAPK: Abcam, ab47363) overnight at 4°C and the secondary antibodies for 2 h at room temperature. After the protein bands were detected by enhanced ECL reagent (BeyoECL Plus, Betyotime, China), the immunoreactive protein bands were quantified by densitometry (Image J software, Wayne Rasband, National Institutes of Health, USA) with a loading control of GAPDH.

### Statistical analysis

All data were expressed as mean ± standard deviation (SD) for three independent tests. SPSS software (Version 17.0) was used to detect statistical difference using the one-way analysis of variance. *P*<0.05 was regarded as a statistically difference.

## Results

### Cell apoptosis ratio

AF cell apoptosis ratio was evaluated by flow cytometry assay. The results showed that in comparison with the control group, high glucose culture significantly increased AF cell apoptosis ratio in a glucose concentration-dependent manner, with a higher apoptosis ratio in the 0.2 M glucose group than that in the 0.1 M group (Figure 1).

**Figure 1:** AF cell apoptosis AF cells among these groups was evaluated by flow cytometry after staining with Annexin V-FITC/PI. Data are expressed as mean ± SD, *n*=3. *: Means a significant difference (*P*<0.05).

### Caspase-3/9 activity

Caspase-3 and caspase-9 are two important mediators in the process of cellular apoptosis. The results showed that high glucose culture obviously increased both caspase-3 activity and caspase-9 activity compared with the control group. Moreover, glucose concentration has a positive relationship with their activity (Figure 2).

**Figure 2:** Caspase-3 and caspase-9 activity of AF cells (**A**) Caspase-3 activity. (**B**) Caspase-9 activity. Data are expressed as mean ± SD, *n*=3. *: Means a significant difference (*P*<0.05).

RETRACTED

### mRNA expression of apoptosis-related molecules

Here, we evaluated mRNA expression of bax, caspase-3 and bcl-2 to assess AF cell apoptosis. The results showed that high glucose culture significantly up-regulated mRNA expression of bax and caspase-3 and down-regulated mRNA expression of bcl-2 compared with the control group. Moreover, these effects of high glucose culture on mRNA expression of these molecules were glucose concentration dependent (Figure 3).

**Figure 3:** Gene expression of apoptosis-related molecules in AF cells Gene expression was analyzed using real-time PCR. Data are expressed as mean ± SD, *n*=3. *: Means a significant difference (*P*<0.05).

### Protein expression of apoptosis markers

In the present study, AF cell apoptosis was also evaluated by analyzing protein expression of two apoptotic markers (cleaved caspase-3 and cleaved PARP). The results showed that high glucose significantly increased protein expression of cleaved caspase-3 and cleaved PARP compared with the control group. Similarly, this also showed a glucose concentration-dependent manner, with a higher expression level in the 0.2 M glucose group than that in the 0.1 M glucose group (Figure 4).

**Figure 4:** Protein expression of apoptosis markers in AF cells (**A**) Images of protein bands. (**B,C**) Gray value analysis of the protein bands of cleaved caspase-3 and cleaved PARP. Protein expression was analyzed using Western blot assay. Data are expressed as mean ± SD, *n*=3. *: Means a significant difference (*P*<0.05).

### Activity of JNK and p38 MAPK pathway

MAPK pathways play an important role in regulating cell activities. Here, we analyzed activity of the JNK pathway and p38 MAPK pathway in AF cells cultured in a high-glucose media. The results showed that a high-glucose media significantly increased protein expression of p-JNK and p-p38 MAPK of AF cells in a glucose concentration-dependent manner (Figure 5).

**Figure 5:** Activity of the JNK pathway and p38 MAPK pathway Their activity was reflected by expression of p-JNK and p-p38 MAPK that was measured by Western blot assay. (**A**) Protein bands and quantitative analysis of p-JNK expression. **(B**) Protein bands and quantitative analysis of p-p38 MAPK expression. Data are expressed as mean ± SD, *n*=3. *: Means a significant difference (*P*<0.05).

### Inhibition of the JNK and p38 MAPK pathway attenuated the effects of high glucose on AF cell apoptosis

Results showed that when the JNK pathway and the p38 MAPK pathway were respectively inhibited by the inhibitor SP600125 and the inhibitor SB203580, the effects of a high glucose (0.2 M) culture on AF cell apoptosis were partly attenuated, which was indicated by the decreased cell apoptosis ratio (Figure 6A) and caspase-3/9 activity (Figure 6B), down-regulated gene or protein expression pro-apoptosis molecules (Bax, caspase-3, cleaved caspase-3 and cleaved PARP) and up-regulated gene expression of anti-apoptosis molecule (Bcl-2, Figure 6C,D).

RETRACTED

**Figure 6:** Inhibition of the JNK pathway and p38 MAPK pathway attenuated AF cell apoptosis (**A**) Apoptosis ratio. (**B**) Caspase-3/9 activity. (**C**) Gene expression of apoptosis-related molecules. (**D**) Protein expression of apoptosis markers. Data are expressed as mean ± SD, *n*=3. *: Means a significant difference (*P*<0.05).

## Discussion

Intervertebral disc degeneration is a common health issue in adults worldwide. Current opinion supports that disc degeneration is a main contributor to lower back pain [2]. Approximately 95% adults experience low back pain at least one time in their lifetime [1]. Cellular apoptosis is a process of programmed cell death which contributes to cellular loss during disc degeneration [22,23]. Decrease in disc cell density and cellular activity will gradually lead to changes in the structure and composition of extracellular matrix since the imbalance between matrix synthesis and degradation [12,24,25]. About twenty years ago, Gruber et al. [22], identified cellular apoptosis in the degenerative human discs. Moreover, disc cell apoptosis is positively related to the degree of disc degeneration [26]. Taking the important role of cell apoptosis in the progression of disc degeneration into account, disc cell apoptosis has become a wide research topic.

DM-associated chronic complications are very complex. Due to the incomplete understanding of the potential etiology of disc degeneration, diabetes is not proved to be a direct risk factor of disc degeneration. Recently, some epidemiological studies have demonstrated that diabetes facilitates disc degeneration, and DM patients have a higher incidence of disc degeneration than non-DM patients [3,27–29]. Several basic researches have investigated the responses of disc cells to high glucose treatment and reported that high glucose significantly promotes senescence of disc NP cells, notochordal cells and AF cells [17–19], and induces apoptosis of disc CEP cells and notochordal cells [20,21]. However, the effects of high glucose on AF cell apoptosis are unclear.

In the present study, we observed the responses of AF cell apoptosis to a high glucose culture. The results showed that compared with the control AF cells, high glucose culture significantly increased cell apoptosis ratio and caspase-3/9 activity, up-regulated mRNA/protein expression of bax, caspase-3, cleaved caspase-3 and cleaved PARP, and down-regulated mRNA expression of bcl-2, indicating that a high glucose culture promotes disc AF cell apoptosis. In addition, our results also showed a positive dose-effect relationship between glucose concentration and AF cell apoptosis. In line with us, several studies also showed that high glucose promotes disc cell apoptosis, such as CEP cells and notochordal cells [20,21]. Hence, inhibiting high glucose-induced disc cell apoptosis may be an effective strategy to retard disc degeneration in DM patients.

RETRACTED

MAPK pathways play an important role in many cell bioactivities, such as cell proliferation, cell senescence and cell apoptosis [30]. Previous studies have showed that the ERK1/2 pathway, p38 MAPK pathway and JNK pathway are associated with disc cell apoptosis under stimulation of certain factors [31–34]. Moreover, these MAPK pathways are also activated under high-glucose conditions in other cells [35,36]. To investigate the signaling pathways behind the effects of high glucose on AF cell apoptosis, we analyzed activity of the JNK pathway and p38 MAPK pathway in AF cells under high-glucose conditions. The results showed that high glucose significantly increased protein expression of p-p38 MAPK and p-JNK in AF cells under high-glucose conditions, indicating that the JNK pathway and p38 MAPK pathway are activated in AF cells under high-glucose conditions. What’s more, we further verify their role in mediating high glucose-induced AF cell apoptosis by using the specific inhibitors. These results provide a possibility that the inhibitor of the JNK pathway or p38 MAPK pathway may be helpful to suppress disc AF cell apoptosis and ultimately play some protective effects against hyperglycemia niche-induced degenerative alterations within the disc AF tissue in DM patient. However, there are lots of work to do to verify their potential clinical application.

The present study also has several limitations. First, rat disc NP tissue contains lots of notochordal cells which may cause cell–cell connection between notochordal cells and AF cells, which is much different from the adult human because notochordal cells are disappeared in adult human disc NP tissue. Second, the present study is just a preliminary study of our research team. Though the present study provides some new information on the effects of hyperglycemia niche on disc AF cell apoptosis in DM patient, we did not further using a DM animal model to further verify our results *in vivo*. Based on our *in vitro* results, we can only speculate that the inhibitor of the JNK pathway or p38 MAPK pathway may have similar inhibitory effects on hyperglycemia niche-induced AF cell apoptosis. However, because the *in vivo* conditions are different from the present *in vitro* simulation, this needs further and systematic investigation.

RETRACTED

## Conclusion

In a word, we observed effects of different concentrations of glucose on AF cell apoptosis. Our results indicate that high glucose significantly promotes disc AF cell apoptosis in a glucose concentration-dependent manner. Through detecting activity of the JNK pathway and p38 MAPK pathway, the present study indirectly suggests that these two pathways may participate in the regulation of high glucose on AF cell apoptosis. The present study provides new knowledge on high glucose-associated disc degeneration, and indirectly suggest that the inhibitor of the JNK pathway or p38 MAPK pathway may be effective in suppressing or retarding disc AF degeneration in DM patient,

## Abbreviations

AF: annulus fibrosus
CEP: cartilage endplate
DM: diabetes mellitus
FITC: fluorescence isothiocyanate
GAPDH: glyceraldehyde-3-phosphate dehydrogenase
JNK: C-Jun NH_2_-terminal kinases
MAPK: mitogen-activated protein kinase
NP: nucleus pulposus
PBS: phosphate buffer solution
PCR: polymerase chain reaction
PI: propidium iodide
PVDF: polyvinylidene fluoride
SD: standard deviation
